# Antibiotic treatment in acute exacerbation of COPD: patient outcomes with amoxicillin vs. amoxicillin/clavulanic acid—data from 43,636 outpatients

**DOI:** 10.1186/s12931-020-01606-7

**Published:** 2021-01-07

**Authors:** Kristian Bagge, Pradeesh Sivapalan, Josefin Eklöf, Frederik Böetius Hertz, Christian Østergaard Andersen, Ejvind Frausing Hansen, Jens Otto Jarløv, Jens-Ulrik Stæhr Jensen

**Affiliations:** 1 Department of Internal Medicine, Respiratory Medicine Section, Herlev and Gentofte Hospital, Copenhagen University Hospital, Hellerup, Denmark; 2 Department of Clinical Microbiology, Hvidovre Hospital, University of Copenhagen, Kettegård Alle 30, 2650 Hvidovre, Denmark; 3 Department of Infectious Diseases, Hvidovre Hospital, University of Copenhagen, Hvidovre, Denmark; 4 Department of Internal Medicine, Zealand University Hospital, Roskilde, Denmark; 5 Department of Clinical Microbiology, Herlev Hospital, University of Copenhagen, Herlev, Denmark; 6 Department of Clinical Microbiology, Slagelse Hospital, Slagelse, Denmark; 7 Department of Internal Medicine, Respiratory Medicine Section, Hvidovre Hospital, University of Copenhagen, Hvidovre, Denmark; 8 Institute for Clinical Medicine, Faculty of Health Sciences, University of Copenhagen, Copenhagen, Denmark

## Abstract

**Background:**

For antibiotic treatment of Acute exacerbations of COPD (AECOPD) the National guidelines in Denmark recommend either first choice amoxicillin 750 mg TID (AMX) or amoxicillin with clavulanic acid 500 mg/125 mg TID (AMC). Addition of clavulanic acid offers a broader spectrum; opposite, AMX alone in a higher dose may offer more time above MIC. The aim of this study was to determine which of these regimens is associated with better outcome.

**Methods:**

The Danish Registry of COPD (DrCOPD), a nationwide outpatient COPD registry, was crosslinked with medication data and hospital contacts. The first prescription of AMX or AMC after inclusion in DrCOPD was used as exposure variable. Adjusted Cox proportional hazards models were used to analyze the risk of hospitalization or death (combined) within 30 days and other endpoints.

**Results:**

For the first treatment of AECOPD 12,915 received AMX, and 30,721 patients received AMC. AMX was associated with a decreased risk of pneumonia hospitalization or death (aHR 0.6, 95% CI 0.5–0.7; p < 0.0001) compared to AMC.

**Conclusion:**

In AECOPD, empirically adding clavulanic acid to amoxicillin is not associated with a better outcome; it seems safe for these patients to be treated with amoxicillin alone.

## Introduction

Acute exacerbations (AECOPD) of chronic obstructive pulmonary disease (COPD) contribute to high morbidity and mortality [1–3]. Key symptoms are breathlessness, increased sputum volume and purulence [4]. The treatment involves the use of bronchodilators, oxygen treatment, systemic corticosteroids and often antibiotics [5]. Antibiotics are used to treat bacterial infections, shorten the course of the disease, prevent further deterioration of lung function, and prolong the period between exacerbations. A quick recovery and longer interval between hospitalizations are important, as both the patient's life and healthcare costs are influenced by the severity and the number of AECOPD [1]. The largest and most recent meta-analysis on treatment of AECOPD [6] concludes in line with earlier meta-analyses [5, 7–9], that for serious exacerbations (requiring hospital admission) there is moderate evidence that antibiotic treatment improves outcomes compared to placebo. For mild to moderate cases (outpatients), the conclusion is less clear, although it is observed, that the risk of treatment failure, defined as no resolution or deterioration of symptoms, is higher among patients who do not receive antibiotics. No effect was found regarding all-cause mortality or re-exacerbations within 2 to 6 weeks. The conclusion was based on pooled data from studies with different antibiotics, and where various doses were used. When using antibiotics, GOLD recommends that the choice is based on local resistance patterns [1]. Today amoxicillin (AMX) 750 mg three times daily (TID) is recommended as first choice empirical treatment of AECOPD in Denmark in mild to moderate cases, however many clinicians prefer amoxicillin with clavulanic acid (AMC) 500/125 mg TID, as recommended in the previous guideline, referring to the fact that AMC is effective against *Moraxella catarrhalis* [10–12]*.* A bacterial pathogen is believed to be accountable for around half of the deteriorations, where *Haemophilus influenzae* are most commonly found, followed by *Streptococcus pneumoniae* and *M. catarrhalis* [13]*.* AMX has a narrow spectrum of activity compared to AMC. Apart from *Staphylococcus aureus* and *M. catarrhalis,* most pathogens that cause community acquired pneumonia and AECOPD that are sensitive to AMC are also sensitive to AMX [14]. The use of AMX instead of AMC in exacerbations in patients with severe COPD has not yet been investigated in a sufficiently large patient population and with clinically important endpoints like pneumonia hospitalization and death. The aim of this study was to determine which of these regimens is associated with better outcomes. On one hand, AMC has a broader spectrum of activity, and on the other hand, AMX is most often administered at a higher dose of amoxicillin (750 mg vs. 500 mg), which may increase the time above the minimal inhibitory concentration (MIC) for many pathogenic bacteria. Additionally, side effects may be more frequent when using AMC [6, 14, 15]. The main analysis compares the risk of death or hospitalization due to pneumonia or AECOPD in the 30 days following a first AMX/AMC prescription.

## Material and methods

This study was designed as a retrospective cohort study. Patients that had at least one hospital outpatient visit were included from the The Danish Registry of COPD [16] (DrCOPD), a nationwide COPD registry. Data were crosslinked with The Danish National Health Service Prescription Database [17], The Danish National Patient Registry [18], a registry of all hospital contacts and The Danish Civil Registration System [19] which includes vital status at any given time. The first prescription of AMX or AMC after inclusion in DrCOPD was used as an exposure variable. The patients were followed for 30 days after they had redeemed a prescription for antibiotics at the pharmacy. Time-to-event data were analyzed using Cox proportional hazards models and expressed as hazard ratios with 95% confidence intervals (CI). The model was adjusted for sex, age, body mass index (BMI), forced expiratory volume in the first second (FEV1), smoking status, prescription of oral corticosteroids ± 7 days from antibiotic prescription, hospitalizations for pneumonia or AECOPD within the past year and comorbidities in form of history of myocardial infarction, heart failure, atrial fibrillation, hypertension, cerebrovascular disease, depression, diabetes, peripheral vascular disease or renal failure. If more than one record of BMI, FEV1 or smoking status existed, the most recent prior to exposure was used. Missing BMI was regarded as a normal value (18.5–24.9), for missing FEV1 and smoking status data, replacement with median values (respectively “30% < FEV1 < 50%” or “Ex-/Non-smoker”) from our data set was performed. All the models were run twice, with these patients included and excluded. Oral corticosteroid prescriptions equal to or below 250 mg prednisolone were classified as short course treatments, prescriptions above 250 mg as long [20]. Comorbidities was based on diagnosis codes from hospital visits in the 10 years prior to inclusion. The primary endpoint was hospitalization for pneumonia or AECOPD (DJ12-DJ18, DJ440 or DJ441), or death by all-cause within 30 days after exposure. Four secondary endpoints were analyzed: (1) time to all-cause hospitalization or death, (2) time to non-pneumonia hospitalization or death, (3) time to death and lastly (4) time to a new prescription of oral antibiotics used for treating lower respiratory tract infections, pneumonia hospitalization or death. For this endpoint moxifloxacin, clarithromycin, roxithromycin, azithromycin, doxycycline, ciprofloxacin, amoxicillin with clavulanic acid and amoxicillin was considered antibiotics used for treating lower respiratory tract infections. It was made as a composite endpoint as to avoid bias i.e. only looking at the mild treatment failures that do not require hospitalization. Microbiological data were available from Region Zealand and the Capital Region of Denmark, accounting for around half of the population in Denmark.

Continuous data were analysed with non-parametric tests (Mann–Whitney-U-test) due to non-normal distributions. Categorical data were compared by using Chi-square or Fischer’s exact tests where appropriate. Multivariable analysis was performed using Cox proportional hazards models while adjusting for the above-mentioned possible confounding variables. Models were controlled for proportional hazards, interactions and linearity. Stratification was performed when appropriate. Comparisons of time-to-event outcomes were summarized via logrank-tests and hazard functions were used for graphic presentations.

A sensitivity analysis was performed by propensity matching our data at baseline by a Greedy matching algorithm [21]. Since there were more patients in the AMC group, they were matched 2 to 1 with the AMX group. All variables included in the primary analysis were used for Greedy matching. For comorbidities, a composite cardiovascular risk factor was made including hypertension, cerebrovascular disease, peripheral vascular disease, atrial fibrillation, heart failure and myocardial infarction. Statistical modelling was performed using SAS 9.4 and R statistical software (V.3.5.2) [22].

## Results

Baseline characteristics are displayed in Table 1. Out of 57,843 patients in the database, 43,639 patients had a prescription for AMX or AMC. Three of these were excluded due to corrupted data. For the first antibiotic treatment, 30,721 received AMC and 12,915 received AMX. Data were complete apart from FEV1 (3691 unknown), BMI (3434 unknown) and smoking group (3701 unknown); the latter were assigned a value as described in the methods (Fig. 1). For age, BMI, FEV1, exacerbations within the past year, prednisolone treatment prescribed along with antibiotics, hypertension, diabetes mellitus and renal failure, before propensity matching, we found a statistical significant difference between the two groups. Microbiological data were available from 2 out of 5 regions in Denmark accounting for around 41% of the patients in our study (Table 2). Eleven percent had a sputum sample examined within 1 week prior to or after starting antibiotic treatment. The distribution of the most common pathogenic bacteria can be seen in Table 3. In our data (273 isolates), we found 81% of *H. influenzae* sensitive to AMX compared to 97% for AMC. Likewise, *M. catarrhalis* is according to EUCAST [23] always reported as resistant to AMX because most strains are slow beta-lactamase producers; this helps explain why in vitro susceptibility testing can be difficult for penicillins with no beta-lactamase inhibitors. Allmost all our isolates were sensitive to AMC.

**Table 1:** Baseline, all patients

	All (43,636)	AMC (30,721)	AMX (12,915)	p-value
Age, median* (IQR)	69 (62–77)	70 (62–77)	69 (61–76)	< 0.0001
Age*				< 0.0001
≤ 62 (Q1)	10,502	7156 (23%)	3346 (26%)	
63–69 (Q2)	9820	6884 (22%)	2936 (23%)	
70–77 (Q3)	12,127	8662 (28%)	3465 (27%)	
≥ 78 (Q4)	11,187	8019 (26%)	3168 (25%)	
Gender female	23,010	16,171 (53%)	6839 (53%)	0.55
FEV1*				< 0.0001
FEV1 ≥ 80%	2289	1438 (5%)	851 (7%)	
50% ≤ FEV1 ≤ 80%	15,778	10,775 (38%)	5003 (43%)	
30% ≤ FEV1 ≤ 50%	14,729	10,659 (38%)	4070 (35%)	
FEV1 ≤ 30%	7149	5416 (19%)	1733 (15%)	
Exacerbations within the past year*	0	24,499 (80%)	11,543 (89%)	< 0.0001
	1	3880 (13%)	902 (7%)	
	≥ 2	2342 (8%)	470 (4%)	
BMI, median* (IQR)	25.0 (21.0–29.0)	24.9 (21.0–29.0)	25.0 (22.0–29.0)	< 0.0001
BMI* (kg/m^2^)				< 0.0001
10.0–18.4	3991	2994 (11%)	997 (8%)	
18.5–24.9	15,763	11,254 (40%)	4509 (38%)	
25.0–29.9	11,823	8252 (29%)	3571 (30%)	
≥ 30	8625	5946 (21%)	2679 (23%)	
Smoking				0.64
Current smokers	14,049	9916 (35%)	4133 (35%)	
Ex-/Non-smokers	25,886	18,329 (65%)	7557 (65%)	
Prednisolone treatment for exacerbation*	No prednisolone	22,290 (73%)	11,692 (91%)	< 0.0001
	Short course treatment	5900 (19%)	979 (8%)	
	Long course treatment	2531 (8%)	244 (2%)	
Comorbidities				
AFLI	3824	2682 (9%)	1142 (9%)	0.71
Heart failure	3399	2422 (8%)	977 (8%)	0.26
Myocardial infarction	2700	1905 (6%)	795 (6%)	0.88
Hypertension*	5800	4001 (13%)	1799 (14%)	0.0113
Diabetes mellitus*	2811	1925 (6%)	886 (7%)	0.0223
Peripheral vascular disease	3843	2684 (9%)	1159 (9%)	0.43
Cerebrovascular disease	3366	2331 (8%)	1035 (8%)	0.13
Renal failure*	989	661 (2%)	328 (3%)	0.0136
Depression	719	514 (2%)	205 (2%)	0.54

^*^ Significant difference found between the two groups (p < 0.05)

**Fig. 1:** Inclusion and exclusion of patients

**Table 2:** Susceptibility testing for key species

Capital region	Susceptibility for AMC Isolates tested (percent sensitive)	Susceptibility for AMX Isolates tested (percent sensitive)
*H. influenzae*	275 (97%)	273 (81%)
*M. catarrhalis*	133 (99%)	^a^
*S. pneumoniae*	109 (100%)	111 (94%)
Other	19 (79%)	53 (25%)

^a^ Should always be reported as R according to EUCAST

**Table 3:** Species distribution in sputum culture from Region Zealand and the Capital Region

	Total	AMC	AMX
Patients included from these regions	17,927	12,481	5446
Sputum sample ± 7 days from inclusion	2012	1821	191
Culture negative	1054	952 (52%)	102 (53%)
*H. influenzae*	353	309 (17%)	44 (23%)
*M. catarrhalis*	178	170 (9%)	8 (4%)
*S. pneumoniae*	152	137 (8%)	15 (8%)
Other^a^	275	253 (14%)	22 (12%)

^a^ Predominantly *Pseudomonas aeruginosa*, enterobacteriaceae and non-haemolytic streptococci

We found that AMX was associated with a decreased risk of pneumonia hospitalization or death by all cause after 30 days compared to AMC (aHR 0.6, 95% CI 0.5–0.7; p < 0.0001; Fig. 2). For secondary endpoints (Fig. 3), we found a weaker association, but still found AMX to be associated with a decreased risk when looking at all-cause hospitalization or death (aHR 0.8, 95% CI 0.8–0.9; p < 0.0001) and non-pneumonia hospitalization or death (aHR 0.9, 95% CI 0.9–1.0; p < 0.0001). When looking at time to a new prescription of antibiotics commonly used for treating lower respiratory tract infections, pneumonia hospitalization or death, we found a slightly increased risk for the patients receiving AMX (aHR 1.2, 95% CI 1.1–1.2; p < 0.0001). When looking only at time to death, we did not find a significant difference (aHR 0.8, 95% CI 0.6–1.0; p = 0.0724).

**Fig. 2:** Pneumonia hospitalization or death

**Fig. 3:** Secondary endpoints

### Sensitivity analysis

As described in the methods, all cox regressions were re-run while excluding all patients with missing values. This did not change the signal of any of the analyses. The model was examined for interaction between antibiotic treatment and exacerbations within the past year (none vs. any). We found a positive interaction (p = 0.0031). Therefore the primary outcome analysis was analyzed within exacerbation strata (0 vs ≥ 1). We found a significant HR below 1.0 for AMX treatment in both groups; though the effect was slightly stronger in the group without any exacerbation, the direction of interpretation was the same for both stratae (i.e. lower risk for amoxicillin treated patients), which were in consequence thereafter presented together.

Additionally, propensity matching was done using the greedy matching algorithm as described in the methods. Baseline data resulting from greedy propensity matching are displayed in Table 4. Of patients treated with AMX, 11,337 were selected and matched with 20,138 patients treated with AMC. Baseline variables seemed well-matched. We found the aHR for pneumonia hospitalization or death on the propensity matched data equal to the original analysis (aHR 0.5; p < 0.0001; Fig. 2).

**Table 4:** Baseline data after propensity matching

	All (31,475)	AMC (20,138)	AMX (11,337)	p-value
Age, median* (IQR)	69 (62–76)	69 (62–77)	69 (61–76)	< 0.0001
Age*				0.0008
≤ 62	7737	4823 (24%)	2914 (26%)	
63–69	7231	4594 (23%)	2637 (23%)	
70–77	8713	5644 (28%)	3069 (27%)	
≥ 78	7794	5077 (25%)	2717 (24%)	
Gender female*	16,431	10,471 (52%)	5960 (53%)	0.33
FEV1*				< 0.0001
FEV1 ≥ 80%	1942	1121 (6%)	821 (7%)	
50% ≤ FEV1 ≤ 80%	12,774	7934 (39%)	4840 (43%)	
30% ≤ FEV1 ≤ 50%	11,661	7671 (38%)	3990 (35%)	
FEV1 ≤ 30%	5098	3412 (17%)	1686 (15%)	
Exacerbations within the past year*	0	17,791 (88%)	10,143 (89%)	0.0028
	1	1601 (8%)	782 (7%)	
	≥ 2	746 (4%)	412 (4%)	
BMI, median* (IQR)	25.0 (21.5–29.0)	25.0 (21.0–29.0)	25.0 (22.0–29.0)	< 0.0001
BMI* (kg/m^2^)				0.0011
10.0–18.4	2810	1853 (9%)	957 (8%)	
18.5–24.9	12,308	7964 (40%)	4344 (38%)	
25.0–29.9	9497	6045 (30%)	3452 (30%)	
≥ 30	6860	4276 (21%)	2584 (23%)	
Smoking*				0.0022
Current smokers	10,802	6787 (34%)	4015 (35%)	
Ex-/Non-smokers	20,673	13,351 (66%)	7322 (65%)	
Prednisolone treatment for exacerbation*	No prednisolone	17,769 (88%)	10,189 (90%)	< 0.0001
	Short course treatment	1899 (9%)	918 (8%)	
	Long course treatment	470 (2%)	230 (2%)	
Comorbidities				
Cardiovascular disease	10,838	6860 (34%)	3978 (35%)	0.07
Diabetes mellitus*	1893	1165 (6%)	728 (6%)	0.0231
Renal failure	682	416 (2%)	266 (2%)	0.11
Depression	453	278 (1%)	175 (2%)	0.26

^*^ Significant difference found between the two groups (p < 0.05)

## Discussion

In this nationwide epidemiological study, we found a pronounced decreased risk of pneumonia hospitalization or death within 30 days (aHR 0.5–0.6 depending on method) in AECOPD outpatients being treated with AMX compared to AMC. This finding was robust to extensive adjustment and was confirmed when the analysis was conducted in a propensity-matched population. One explanation for our findings might be the dosing of antibiotics. The serum profile of the amoxicillin component is the same, when administered with and without clavulanic acid [10, 24], thus it would be very unlikely that AMC is inferior to AMX when administered in equal doses. A study group measured AMX in sputum samples from 33 hospitalized AECOPD patients treated with AMC and found longer hospitalization (7 vs 11 days) when AMX concentrations did not reach target (2 mg/L) [25]. Two third of their patients did not reach target in sputum. In another study by the same group [26] with 23 hospitalized AECOPD patients 78% of the patients did not reach target in sputum. Oral (500 mg TID/QID) vs intravenously (1000 mg QID) administration was highly associated with the likelihood of reaching target sputum concentration. The lower amoxicillin concentration in sputum did not seem to interfere with the efficacy. AMC is usually and as per Danish guidelines administered 500/125 mg TID whereas AMX per guideline is administered 750 mg TID, and often dosed higher such as 1 g TID or QID. AMX and AMC exhibit time dependent killing [27] and the efficacy of the compounds depends on the time where the antibiotic concentration is higher than MIC (T > MIC) at the site of infection [14, 27]. For betalactam antibiotics to be efficient against *S. pneumoniae* and *H. influenzae,* T > MIC should be greater than 40% [10, 27, 28]. When pathogens are sensitive to AMX, such as most *S. pneumoniae* and *H. influenzae,* it is the concentration of the AMX component that determines the efficacy for threatment with AMC [10]. The different doses of the AMX component in our population (500 mg vs 750 mg TID) might influence T > MIC sufficiently to affect efficacy. According to monte carlo simulations [28], the dose of 500 mg TID amoxicillin should be sufficient for most pathogens. The optimal combination and dose of each constituent in AMC have been debated through time, and more evidence is still needed as to what combinations give the best efficacy and lowest rate of side effects [10, 14]. Another contributing factor could be toxicity from broad-spectrum antibiotics like AMC. In a recent meta-analysis of randomized controlled trials assessing the clinical outcomes in patients treated with an antibiotic-sparing biomarker-guided regimen as compared to standard care it was observed, apart from a pronounced reduction in the use of antibiotics, that such an antibiotic reduction did actually lead to a significantly lower mortality and fewer adverse antibiotic effects [29].

The most important limitation to our study is the risk of residual confounding by indication since AMC could be given generally to patients in worse condition. At baseline, we did find differences between the two groups regarding some variables; however, this seemed to be fairly well evened out after propensity matching. Although we did our utmost to match and adjust for known confounders, we cannot rule out some residual confounding by indication. We did find a positive interaction between the antibiotic treatment (AMX/AMC) and the number of hospitalizations due to pneumonia or AECOPD within the past year (none vs any) toward the primary outcome. However, when we stratified the data and analyzed these two stratae separately, we found that the HR for AMX treated patients was significant and below 1.0 for both and thus, by and large, the signal was not different (lower risk in AMX-treated patients). Another limitation is, that we did not know any acute physical measures for AECOPD severity; however, none of these patients had severe exacerbations as they were not admitted to a hospital. As concerns antibiotic dosing, though we did know the formulation and the quantity prescribed, we did not know daily dose instructions or patient compliance. However, since guidelines exist for both AMX and AMC prescriptions in AECOPD, it is likely that most instructions are made accordingly. Finally, the indication leading to antibiotic prescription was not available. Although it is likely that some of the AMX/AMC prescriptions were made for indications other than AECOPD, we think it is unlikely that the proportions of AMX and AMC prescribed for non-AECOPD differ much. In Denmark, neither AMX or AMC is usually used for empirical treatment of UTI.

In our secondary outcome analysis (all-cause hospitalization and non-pneumonia hospitalization) we observed aHR for AMX close to 1.0 (and thus not as low as for the primary outcome of pneumonia hospitalization or death), which argues that confounding by indication cannot explain our main results. Had this been the case, we would expect the aHR to be low for most of the unfavourable outcomes. Our analysis of need for additional antibiotics, pneumonia hospitalization or death showed an aHR of 1.2. It is important to keep in mind, that some of the new prescriptions being made is secondary to findings by cultivation and does not necessarily represent a clinical treatment failure. This is more likely to happen when treating with amoxicillin without beta-lactamase inhibitor. The result of this analysis should thereby be read with caution. When looking at death only, we see a broad CI (0.6–1.0) and few incidents, indicating that the combined endpoint pneumonia hospitalization or death is primarily driven by pneumonia.

Few studies compare the use of AMX instead of AMC in AECOPD, without also looking at other antibiotics at the same time in a small-spectred vs. broad-spectred analysis. We identified one article [30] that directly compares AMX with AMC in AECOPD. It was conducted prospectively in 137 patients in an outpatient setting and did not find any difference in outcome (clinical cure assessed by a physical examination on day 10 and 30). The study population did not have as advanced COPD as in our population, and there was no information on hospitalization or death.

Overall we find no indication in our data, that treatment with AMX is inferior to AMC. There is a need to avoid the use of broad-spectrum antibiotics to reduce the risk of selecting resistant strains and to cause least possible side effects and dysregulation in the patient´s microbiome. This study supports the use of AMX as first choice antibiotic treatment in non-hospitalized patients suffering from AECOPD.

## Conclusion

In AECOPD, treatment with AMX 750 mg TID was associated with substantially better outcomes than AMC 500/125 mg TID within 30 days. Reasons may include under-dosing of amoxicillin with AMC and residual confounding by indication.

## Data Availability

The datasets analysed during the current study are not publicly available due to the Danish Data Protection Act, but are available from the corresponding author on reasonable request, after approval has been given by the Danish Data Protection Agency.
